This article has been retracted.

# Exosome-Delivered LncHEIH Promotes Gastric Cancer Progression by Upregulating EZH2 and Stimulating Methylation of the GSDME Promoter

**DOI:** 10.3389/fcell.2020.571297

**Published:** 2020-10-14

**Authors:** Yan Lu, Kaiqing Hou, Mengsen Li, Xiaobin Wu, Shaochun Yuan

**Affiliations:** ^1^Guangdong Province Key Laboratory of Pharmaceutical Functional Genes, Key Laboratory of Gene Engineering of the Ministry of Education, College of Life Sciences, Sun Yat-sen University, Guangzhou, China; ^2^Department of Gastrointestinal Surgery, The 8th Affiliated Hospital of Sun Yat-sen University, Shenzhen, China; ^3^Hainan Provincial Key Laboratory of Carcinogenesis and Intervention, Hainan Medical College, Haikou, China; ^4^Department of Gastrointestinal Surgery, Haikou City People’s Hospital, Haikou, China

**Keywords:** exosome, lncHEIH, EZH2, GSDME, gastric cancer

## Abstract

Gastric cancer is the third leading cause of cancer-related deaths worldwide and is characterized by poor survival and high recurrence rates. Long non-coding RNAs (lncRNAs) have gained considerable attention in recent years as prognostic markers and gene regulators in various cancers. Here, we found that lncHEIH was upregulated in gastric cancer tissues and cell lines and positively correlated with high expression levels of EZH2. Mechanistically, the lncHEIH-EZH2 axis could promote the progression of gastric cancer. In addition, lncHEIH encapsulated in exosomes was released by gastric cancer cells and then absorbed by normal gastric cells. The uptake of lncHEIH resulted in the upregulation of EZH2, which inhibited the expression of the tumor suppressor GSDME by methylation of the GSDME promoter, promoting the malignant transformation of normal gastric cells. Overall, lncHEIH promotes gastric cancer progression by upregulating the expression of EZH2 and reducing the expression of GSDME in normal cells to induce malignant cell proliferation and migration, indicating its potential as a target in gastric cancer therapy.

## Introduction

Gastric cancer is the fifth most common malignancy and the third leading cause of cancer-related mortality worldwide (Enjoji et al., 2018; Ferlay et al., 2019). It is responsible for 800,000 deaths every year, and one million new patients are diagnosed annually (Jemal et al., 2011; Rebecca et al., 2018; Ferlay et al., 2019). However, the mechanisms underlying the initiation and development of gastric cancer remain largely elusive. In recent years, the role of the tumor microenvironment in promoting gastric cancer progression has gained considerable attention (Kenny et al., 2007). The tumor microenvironment is a complex system that includes cancer stem cells (CSCs), immune cells, fibroblasts, blood vessels, exosomes, and secreted inflammatory cytokines and is a key factor involved in tumor growth and metastasis (Wu and Dai, 2017; Barbora et al., 2019).

Exosomes in the tumor microenvironment are small vesicles secreted from cells that mediate signal transduction between neighboring or distant cells (Thery et al., 2002; Cocucci et al., 2009), which regulate the tumor microenvironment by paracrine means (Kahlert and Kalluri, 2013; Chan et al., 2015). Exosomes transport essential cargo such as proteins, lipids and nucleic acids, including microRNAs (miRNAs), circular RNAs and long non-coding RNAs (lncRNAs) (Skog et al., 2008; Lai et al., 2010). Exosomal lncRNAs and their roles in cancer have gained considerable attention in recent years, such as lncH19, UCA1 and PCAT1 which can be encapsulated in plasma-derived exosomes (Li et al., 2015; Zhang et al., 2019). LncHEIH was located on chromosome 5 with a length of 1652 bp, first discovered in hepatocellular carcinoma (HCC) and then shown to be highly expressed in colorectal cancer (CRC) (Yang et al., 2011; Cui et al., 2018). However, the expression pattern of lncHEIH in gastric cancer is still unclear.

The role of lncHEIH in cancer progression is mediated by binding to the EZH2 subunit of the PRC2 complex to regulate the expression of several target genes (Yang et al., 2011). EZH2 is a critical component of the PRC2 complex, which plays an essential role in the progression of cancer (Benetatos et al., 2013; Luo et al., 2013). EZH2 is frequently overexpressed in various cancers and is a critical molecule for promoting the proliferation of cancer cells, tumorigenesis and CSC maintenance (Yamagishi and Uchimaru, 2017). As reported, EZH2 is upregulated in the CSC of various malignant tumors, such as melanoma cancer, breast cancer, ovarian cancer, and CRC (Liu et al., 2014; Tiffen et al., 2015).

GSDME (also named DFNA5) is a key pyroptotic substrate of caspase. The methylation level of the GSDME promoter is 65% in CRC tissue but only 3% in normal colorectal tissue (Kim et al., 2008). Similar results were found in breast cancer (Fujikane et al., 2010). This evidence implies that high methylation of the GSDME promoter is a pivotal factor for blocking the expression of GSDME, leading to an impaired role of GSDME in suppressing tumorigenesis. However, the mechanisms of GSDME promoter methylation are not well-understood.

To reveal the role of the lncHEIH-EZH2 axis in gastric cancer and shed some light on the downregulation of GSDME, we first detected high endogenous levels of lncHEIH in gastric cancer tissues compared to normal tissues. Similar to other observations, ectopic expression of lncHEIH promoted gastric cancer progression. Furthermore, lncHEIH could be released by gastric cancer cells through exosomes, which were subsequently taken up by normal gastric cells, resulting in the malignant proliferation and metastasis of normal cells via upregulation of EZH2 and downregulation of the tumor suppressor gene GSDME. Our results highlight the important role of lncHEIH in promoting gastric cancer progression, indicating its potential as a target in gastric cancer therapy.

## Materials and Methods

### Tissue Samples

Human gastric cancer tissues and paired adjacent non-cancerous tissues were collected from patients who underwent surgical resection at the Sixth Affiliated Hospital of Sun Yat-sen University between December 2016 and August 2018. Out of a total of 21 patients, 15 were men and 6 were women, with an average age of 60.9 (range: 39–79) years. The study protocol was approved by the Sun Yat-sen University Institutional Animal Care and Use Committee. Written informed consents were obtained from all participants.

### Cell Lines and Reagents

Primary gastric cancer cells were established from tumor tissues as previously described (Herrera et al., 2016) and maintained in DMEM/F12 (Gibco) supplemented with 10% foetal bovine serum (FBS), 100 μg/ml streptomycin and 100 U/ml penicillin. The gastric cell lines AGS, HGC-27 and GES-1 were maintained in our lab and cultured at 37°C in an atmosphere containing 5% CO_2_ in DMEM supplemented with 10% FBS. The cell lines were authenticated by 16-loci short tandem repeat (STR) profiling in October 2018.

### Cell Proliferation Assays

Cell proliferation was evaluated by the ethynyl deoxyuridine (EdU) incorporation assay and CCK-8 assay using the BeyoClick EdU Cell Proliferation Kit (Beyotime) and Cell Counting Kit-8 Assay Kit (Beyotime) according to the manufacturer’s instructions. Briefly, the cells were seeded in 24-well plates and transfected with 1 μg suitable vectors or 50 nmol/L siRNAs, after which the assay was performed. The actively proliferating EdU-positive cells were detected by stereomicroscopy and their percentage was calculated by flow cytometry. For the CCK-8 assay, transfected cells were seeded in 96-well plates at a density of 2 × 10^3^ cells/well and then maintained in 10% FBS DMEM for 24, 48, and 72 h. Cell viability was evaluated by the Enhanced Cell Counting Kit-8 at each time point. The absorbance was measured at 450 nm by a microplate reader. Experiments were repeated at least three times.

### Cell Migration

Cell migration assays were performed in 24-well Transwell chambers (Corning) as previously described (Zhu et al., 2017). The cells were seeded into the upper chambers in serum-free DMEM at a density of 1 × 10^5^ cells per well, and 200 μl sterile complete DMEM (with 20% FBS) was dispensed into the lower chambers as the chemoattractant. After 24 h, the migrated cells on the lower surface of the filters were fixed in 4% paraformaldehyde (Sangon Biotech) for 10 min and stained with crystal violet (Beyotime) for 10 min at room temperature. The number of migrated cells was counted in five non-overlapping fields under a stereomicroscope (Leica Microsystems CMS GmbH). Experiments were repeated at least three times.

### Xenograft Tumor Model

Xenograft experiments were performed as previously described (Zhu et al., 2017). All studies were approved by the Sun Yat-sen University Institutional Animal Care and Use Committee. Briefly, HGC-27 cells stably transfected with sh-lncHEIH or sh-ctrl were harvested, and 1 × 10^7^ cells/mouse were subcutaneously injected into a single side of 4-week-old female athymic nude mice (provided by Experimental Animal Center of Guangdong Province). Tumor sizes were measured by calipers every 3 days. The tumor volumes were calculated from the length and width using the following formula: π/6 × length × width^2^ (Chen et al., 2018). The mice were killed after 20 days, and the tumors were resected and fixed in formaldehyde for further assays.

### Flow Cytometry

The indicated cells were seeded into 24-well plates at a density of 5 × 10^3^ cells/well, transfected with 1 μg suitable vectors, and harvested cells 48 h later using trypsin. The cells were resuspended in PBS and stained with FITC-conjugated anti-human CD44 (eBioscience) and APC-conjugated anti-human EPCAM (eBioscience) antibodies as previously described (Lau et al., 2014). The stained cells were detected using a FACSCalibur (Beckman CytoFLEX FCM). Experiments were repeated at least three times.

### Exosome Isolation and Characterization

Exosomes released by gastric cancer cells were isolated from serum-free medium by differential centrifugation. The supernatant fluid was centrifuged at 500 *g* for 10 min to eliminate cells and ultracentrifuged at 120,000 *g* for 70 min to pellet the exosomes. The pellet was washed in PBS to eliminate impurity proteins, and centrifuged again at 120,000 *g* for 70 min. The PBS was removed and the exosomes were re-suspended in 100 μl PBS (Valadi et al., 2007). The specific exosomal protein markers were determined by Western blotting, and the morphological assessment was made by electron microscopy. Total RNA from exosomes and serum-free media was isolated using an exoRNeasy Serum/Plasma Starter Kit (Qiagen) according to the manufacturer’s instructions.

### Western Blotting

The cells were lysed in RIPA lysis buffer (Beyotime) supplemented with 1 mM PMSF for 30 min on ice. Total protein was separated by 10% SDS-PAGE, transferred to NC membranes, and probed with antibodies against human EZH2 (66476-1-Ig, Proteintech), GSDME (13075-1-AP, Proteintech), CD9 (20597-1-AP, Proteintech), CD63 (25682-1-AP, Proteintech), Calnexin (66903-1-Ig, Proteintech), CD81 (sc-7637, Santa Cruz), PTEN (22034-1-AP, Proteintech), and GAPDH (10494-1-AP, Proteintech). Peroxidase-conjugated anti-mouse and anti-rabbit secondary antibodies (Proteintech) were used to probe the positive bands, which were visualized by enhanced chemiluminescence assay (ECL, Millipore). In western blotting analysis, antibody dilutions were 1:1000 for EZH2, GSDME, CD9, CD63, Calnexin, CD81 and PTEN, 1:5000 for GAPDH and secondary antibodies. Experiments were repeated at least three times.

### Quantitative Real-Time PCR (qRT-PCR) Assay

Total RNA was isolated using TRIzol (Invitrogen) or RNeasy kit (QIAGEN) according to the manufacturer’s instructions and reverse transcribed into cDNA using Prime Script RT reagent Kit with gDNA Eraser (TAKARA) and random primers (TAKARA). qRT-PCR was performed on a Roche Real-Time PCR System (Roche Light Cycler 480II), and the expression data of specific genes were normalized to GAPDH expression or to control samples data. Primers sequences were as follows: primers for lncHEIH (forward: 5′-CCTCTTGTGCCCCTTTCT-3′; reverse: 5′-AGGTCTCATGGCTTCTCG-3′), primers for EZH2 (forward: 5′-AATCAGAGTACATGCGACTGAGA-3′; reverse: 5′-GCTGTATCCTTCGCTGTTTCC-3′), primers for EPHB3 (forward: 5′-TGGGTAACATCTGAGTTGGCG-3′; reverse: 5′-TGGTATGTGCGGATGGGATTC-3′), primers for E-cadherin (forward: 5′-GGTCTGTCATGGAAGGTGCT-3′; reverse: 5′-CGTAGGGAAACTCTCTCGGTC-3′), primers for STAT3 (forward: 5′-CAGCAGCTTGACACACGGTA-3′; reverse: 5′-AAACACCAAAGTGGCATGTGA-3′), primers for P16 (INK4A) (forward: 5′-GTGAGAGTGGCGGGGTC-3′; reverse: 5′-GTTACGGTCGGAGGCCG-3′), primers for GSDME (forward: 5′-ATTCTGGTGCTGGCAGAGAC-3′; reverse: 5′-GTTCCACTCACGTGGTTTGC-3′), primers for GSDMB (forward: 5′-TCCTGATTTCCGGGGAGCTA-3′; reverse: 5′-CCAAGACCCCAGCAGCATTA-3′), primers for PTEN (forward: 5′-CACCTATTCCTCAGCCCTTAT-3′; reverse: 5′-AACCCTCATTCAGACCTTCAC-3′); and primers for GAPDH (forward: 5′-ACGGGAAGCTTGTCATCAAT-3′; reverse: 5′-TGG ACTCCACGACGTACTCA-3′).

### Transfection and Selection of Stable Cell Lines

HGC-27 cells seeded in 6-well plates were transfected with 2 μg shRNAs against lncHEIH or scrambled shRNAs using Lipofectamine 3000 (Invitrogen) in Opti-MEM serum-free medium according to the manufacturer’s protocol, and stably transfected cells were selected with puromycin (1.5 μg/ml) for 2 weeks. For siRNAs transfection, the cells were plated in a 12-well plate at a density of 1 × 10^5^ cells/well and transfected 50 nmol/L siRNA into cells using Lipofectamine 3000 (Invitrogen) according to the manufacturer’s instructions. Experiments were routinely performed in triplicate wells and repeated at least three times. The siRNAs were obtained from Sangon Biotech, Co., Ltd. (Shanghai, China). The sequences of siRNAs and shRNAs were as follows: sense of si-lncHEIH1 5′-GCGCCUUCCCUCUAACCUUAA-3′; sense of si-lncHEIH2 5′-GGCAAGAUGAACGUCUGAAAU-3′; sense of si-EZH2-1 5′-GAUAGAGAAUGUGGGUUUA-3′; sense of si-EZH2-2 5′-GGAUGGUACUUUCAUUGAA-3′; shRNA-HEIH-1: 5′-TGCGCCTTCCCTCTAACCTTAATT CAAGAGATTAAGGTTAGAGGGAAGGCGCTTTTTTC-3′; and shRNA-HEIH-2: 5′-TGGCAAGATGAACGTCTGAAA TTTCAAGAGAATTTCAGACGTTCATCTTGCCTTTTTTC-3′.

### Oncosphere Formation Assay

Oncospheres were generated as previously described (Wang et al., 2015). Briefly, primary gastric cancer cells (1000 cells per pore) were seeded on ultra-low attachment culture dishes (Corning) in serum-free DMEM/F12 (Invitrogen) containing 2 mM L-glutamine, 1% sodium pyruvate (Invitrogen), 100 μg/ml penicillin and 100 U/ml streptomycin, supplemented with 20 ng/ml epithelial growth factor (Invitrogen), 10 ng/ml fibroblast growth factor-2 (Invitrogen) and B27 (Invitrogen). The cells were cultured in suspension for 10 days. The number of oncospheres with diameters > 75 μm was counted under a stereomicroscope (Leica Microsystems CMS GmbH). Oncospheres were harvested using 70 μm cell strainers and dissociated into single cells with trypsin, after which the number of cells in each oncosphere was counted (Sendurai et al., 2008).

### Immunohistochemistry (IHC) Assay

The tumors resected from the nude mice were fixed in paraformaldehyde and processed according to standard protocols. The tissue sections were probed for the specific marker EZH2 using IHC according to standard protocols as previously described (Zhu et al., 2017).

### Luciferase Reporter Assay

HEK293T cells seeded in 48-well cell culture plates were transfected with 100 ng of the luciferase reporter vector containing the human GSDME promoter together with the EZH2 expression vector or empty control plasmid. A total of 10 ng of Renilla luciferase reporter gene vector was transfected simultaneously as an internal control. After 24 h, the luciferase activity was measured with the Dual Luciferase Reporter Assay System (Promega). Experiments were routinely performed in triplicate wells and repeated at least three times.

### Methylated Bisulfite Sequencing PCR

GES-1 cells were seeded in the 12-well plate format at approximately 70% confluency and transfected with 1 μg pEZ-EZH2 or empty control plasmid. Genomic DNA was isolated using the Ezup Column Animal Genomic DNA Purification Kit (Sangon Biotech) according to the manufacturer’s instructions. Bisulfite treatment of DNA and bisulfite genomic sequencing PCR were carried out as previously described (Owa et al., 2018). PCR products were cloned into the pUC18 vector using T4 DNA Ligase (TAKARA). Then, the PCR products were sequenced and analyzed. Bisulfite sequencing PCR was performed by Sangon Biotech, Co., Ltd. The primers used were as follows: F: 5′-ATAGGTTTTGGATTTTTTTGGTT-3′; R: 5′-CCAAAAACCCCAAAAAAAAC-3′.

### Statistical Analyses

All quantitative data are presented as the mean ± SD of at least three independent experiments. All the statistical analyses were performed using SPSS 13.0 (SPSS, United States). The Student’s *t*-test was used to compare the statistical significance between two groups by SPSS 13.0 and GraphPad Prism (GraphPad Software, United States). *P*-values < 0.05 were considered statistically significant.

## Results

### Upregulated LncHEIH in Gastric Cancer Promotes Proliferation and Migration of Gastric Cancer Cells

Although lncHEIH has been reported to be upregulated in HCC and CRC, the expression of lncHEIH in gastric cancer is unknown. To explore whether lncHEIH was upregulated in gastric cancer, we determined lncHEIH expression by qRT-PCR. The results showed that the transcription level of lncHEIH was significantly higher in gastric cancer tissues than in adjacent normal tissues (Figure 1A), and it was also higher in primary gastric cancer cells (established from fresh tumor tissues and identified as typical epithelial cells in Figure 1B) and immortalized gastric cancer cells (AGS and HGC-27) than in normal gastric epithelial GES-1 cells (Figure 1C).

**FIGURE 1:** Upregulated lncHEIH in gastric cancer promotes the proliferation and migration of gastric cancer cells. **(A)** Median lncHEIH expression levels in 21 paired gastric cancer and adjacent normal tissues. **(B)** Primary gastric cancer cells established from fresh tumor tissues were identified by immunofluorescence. The green fluorescence indicates cytokeratin-19, and the red fluorescence indicates vimentin. **(C)** Relative lncHEIH levels in the GES-1, AGS, HGC-27 cell lines and primary gastric cancer cells normalized to GAPDH levels. The results are shown as the mean ± standard deviation from three independent experiments. **(D,E)** LncHEIH levels in gastric cancer cells transfected with lncHEIH or si-lncHEIH for 48 h. **(F)** Representative images showing the EdU^+^ proliferating gastric cancer cells transfected with lncHEIH or si-lncHEIH for 48 h. The red color indicates EdU^+^ nuclei (scale bars = 50 μm). **(G)** Graphs showing the proportion of EdU^+^ cells in different groups detected by flow cytometry. **(H)** Representative images of the Transwell assay showing the migration of gastric cancer cells transfected with lncHEIH or si-lncHEIH (scale bars = 50 μm). **(I)** Bar graph showing the number of migrated cells. The results shown are the mean ± SD from three independent experiments. *P < 0.05, **P < 0.01, ***P < 0.001.

To determine the biological role of lncHEIH in stimulating the progression of gastric cancer, primary gastric cancer cells and HGC-27 cells were transfected with either pcDNA3.1-HEIH or si-lncHEIH (Figures 1D,E). The EdU incorporation assay showed a significant increase in the proportion of EdU^+^ proliferating cells transfected with the lncHEIH expression vector, whereas lncHEIH knockdown generated the opposite results (Figures 1F,G). Furthermore, Transwell assays showed that overexpression of lncHEIH significantly increased the migratory capacity of gastric cancer cells, while silencing the expression of lncHEIH significantly decreased the numbers of migratory gastric cells *in vitro* (Figures 1H,I). Overall, lncHEIH enhances the proliferation and migration of gastric cancer cells.

### LncHEIH Enhances Tumorigenesis of Gastric Cancer Cells and the Expansion of Gastric CSC

To validate the effect of lncHEIH *in vivo*, HGC-27 cells were stably transfected with either scrambled or lncHEIH-targeting shRNA. Then, the cells were inoculated into nude mice, and subcutaneous tumor xenografts were regularly monitored. The results indicated that knockdown of lncHEIH expression significantly inhibited tumorigenesis and reduced tumor weight and size compared to the control xenografts (Figures 2A–C). The expression level of lncHEIH in the harvested tumors was consistent with its expression status in the respective HGC-27 inocula (Figure 2D).

**FIGURE 2:** LncHEIH promotes *in vivo* tumorigenesis of gastric cancer cells and expansion of gastric CSC. **(A)** HGC-27 cells transfected with Ctrl shRNA or lncHEIH shRNA were injected into nude mice (*n* = 5), which were killed by carbon dioxide euthanasia 20 days after injection. **(B)** Tumor volumes were calculated every 3 days starting at 5 days after injection. Bars indicate SD. **(C)** Tumor weights are represented as the mean tumor weights ± SD. **(D)** The expression level of lncHEIH in the harvested tumors was tested by qRT-PCR. **(E,F)** The percentage of CD44^+^EPCAM^+^ CSC among primary gastric cancer cells transfected with lncHEIH. **(G,H)** Representative images of oncospheres formed by primary gastric cancer cells cultured in serum-free spheroid suspension culture for 10 days and the number of spheres per 1000 cells (scale bar = 100 μm). **(I,J)** Representative image of oncospheres and the number of cells per sphere after 10 days (scale bar = 50 μm). Error bars denote ± SD. *P < 0.05, **P < 0.01, ***P < 0.001.

Recent studies have shown that lncRNAs promote tumor malignant transformation by stimulating CSC expansion (Wang et al., 2015). Therefore, the proportion of EpCAM^+^/CD44^+^ gastric CSC was measured. Unsurprisingly, flow cytometry assay results displayed a significant increase in the proportion of CSC among lncHEIH-overexpressing primary gastric cancer cells (Figures 2E,F). To further determine the potential role of lncHEIH in gastric CSC, we evaluated the self-renewal ability of primary gastric cancer cells by an *in vitro* oncosphere formation assay. As shown in Figures 2G,H, overexpression of lncHEIH significantly enhanced the number of oncospheres compared to that in the control cells. Furthermore, the oncospheres overexpressing lncHEIH were larger and contained 2.5-fold more cells per sphere relative to the control (Figures 2I,J). Taken together, the results demonstrate that lncHEIH enhances the tumorigenicity of cancer cells and the expansion of gastric CSC.

### LncHEIH Promotes Gastric Cancer Progression by Upregulating EZH2

Although the above evidence confirms that lncHEIH could promote the progression of gastric cancer, the molecular mechanism remains unclear. Since lncHEIH is known to bind to EZH2, we analyzed the expression of EZH2 and found a significant positive correlation between the *in situ* expression levels of lncHEIH and EZH2 mRNA in the paired gastric cancer tissues (Figure 3A). Furthermore, the EZH2 expression levels were significantly higher in tumors derived from control cells than lncHEIH-knockdown HGC-27 cells (Figure 3B). In addition, the expression of EZH2 was significantly enhanced when lncHEIH was overexpressed in the primary and immortalized gastric cancer cell lines. Conversely, knockdown of lncHEIH had the opposite effect (Figure 3C). To determine whether lncHEIH functions upstream of EZH2 in the regulation of gastric cancer proliferation, migration and CSC expansion, we silenced EZH2 in lncHEIH-overexpressing primary gastric cancer cells. Since the time of stem cell spheroidization is about 10 days, we tested the interference effect of EZH2 at 48 h and 10th day (Figure 3D). Interestingly, the silencing of EZH2 reduced the proliferation, migration and oncosphere formation ability of gastric cancer cells (Figures 3E–K). These results indicated that lncHEIH promotes gastric cancer progression by upregulating EZH2.

**FIGURE 3:** LncHEIH promotes gastric cancer progression by upregulating EZH2. **(A)** LncHEIH and EZH2 mRNA levels in paired gastric cancer tissue samples and correlation analysis. Data were normalized to GAPDH expression. **(B)** The tumor sections were subjected to IHC staining using antibodies against EZH2 (scale bars = 50 μm). **(C)** Immunoblot showing EZH2 protein levels in gastric cancer cells transfected with lncHEIH or si-lncHEIH for 48 h. **(D)** EZH2 mRNA levels in primary gastric cancer cells transfected with siEZH2. **(E)** CCK-8 analysis determined the viability of primary gastric cancer cells transfected with lncHEIH and siEZH2-2. **(F,G)** Transwell assays were used to determine the migration ability of primary gastric cancer cells transfected with lncHEIH and siEZH2-2 (scale bars = 50 μm). **(H,I)** Percentage of CD44^+^ EPCAM^+^ CSC among primary gastric cancer cells transfected with lncHEIH and siEZH2-2. **(J,K)** Representative image of oncospheres and the number of cells per sphere after 10 days (scale bar = 50 μm). Data are shown as the mean ± SD. *P < 0.05, **P < 0.01, ***P < 0.001.

### LncHEIH Encapsulated in Exosomes Can Be Released Extracellularly by Gastric Cancer Cells

Studies have shown that lncRNAs can be transferred from donor cells to distant locations via extracellular vesicles such as exosomes (Fan et al., 2018; Sun et al., 2018; Zheng et al., 2018). In HCV-related hepatocellular carcinoma, lncHEIH can be transported into the blood by exosomes (Zhang et al., 2018). To determine whether lncHEIH can be transported similarly in gastric cancer, we extracted exosomes from the culture supernatant of gastric cancer cells. The exosomes were characterized by morphology (Figure 4A) and the basis of surface expression of CD63, CD9, and CD81. Calnexin was used as a negative control based on its low endogenous expression in exosomes (Figure 4B). The detection of lncHEIH in the exosomes and cell culture medium suggested that lncHEIH encapsulated in exosomes can be released extracellularly by gastric cancer cells (Figure 4C).

**FIGURE 4:** LncHEIH encapsulated in exosomes can be released extracellularly by gastric cancer cells and enter normal cells. **(A)** Electron scanning microscopy of exosomes released by gastric cancer cells (scale bar = 200 nm). **(B)** Immunoblot showing the protein levels of CD63, CD9, CD81, and Calnexin in the isolated exosomes. **(C)** LncHEIH mRNA levels in exosomes (from 20 ml serum-free medium) and 20 ml serum-free medium. **(D)** LncHEIH levels in cells and exosomes when gastric cancer cells were transfected with shHEIH-2 and cultured in serum-free medium. **(E)** LncHEIH mRNA levels in GES-1 cells when exosomes and shHEIH-exosomes were added to the cultures for 48 h. Data are shown as the means ± SD. The images are representative of three independent experiments. *P < 0.05, **P < 0.01, ***P < 0.001.

### Exosome-Delivered LncHEIH Promotes the Proliferation and Metastasis of Normal Gastric Cells Through the LncHEIH-EZH2 Axis

To determine the biological function of exosome-delivered lncHEIH, we first isolated exosomes secreted by control and lncHEIH-knockdown HGC-27 cells. Then, the expression level of lncHEIH in both cell line and exosomes was validated (Figure 4D). After incubating the exosomes with GES-1 cells (5 μg exosomes per 5 × 10^5^ cells), the uptake of exosome-delivered lncHEIH was detected by qRT-PCR (Figure 4E). Then, the ethynyl deoxyuridine (EdU) incorporation assay, CCK-8 assay and Transwell assay were performed to detect the effect of exosome-delivered lncHEIH on cell proliferation and migration. The results showed that exosomes containing lncHEIH significantly promoted the proliferation and migration of GES-1 cells (Figures 5A–E). Furthermore, we found that in normal gastric cells, the expression of EZH2 was significantly enhanced when lncHEIH was overexpressed or exosomes containing lncHEIH were added (Figure 5F). Next, to investigate whether the role of lncHEIH in normal gastric cells is related to the lncHEIH-EZH2 axis, we silenced EZH2 in the lncHEIH-overexpressing normal gastric cell line GES-1. The silencing of EZH2 reduced the malignant proliferation and migration ability affected by lncHEIH (Figures 5G–I). Therefore, exosome-delivered lncHEIH promotes the proliferation and metastasis of normal gastric cells through the lncHEIH-EZH2 axis.

**FIGURE 5:** Exosome-delivered lncHEIH promotes the proliferation and metastasis of normal gastric cells by the lncHEIH-EZH2 axis. **(A)** Representative images showing the EdU^+^ proliferating GES-1 normal gastric cells transfected with lncHEIH or added exosomes to the medium for 48 h. The red color indicates EdU^+^ nuclei. Scale bars = 50 μm. **(B)** Graphs showing the proportion of EdU^+^ cells in different groups detected by flow cytometry. **(C)** CCK-8 analysis was used to determine the viability of GES-1 cells transfected with lncHEIH or added exosomes to the medium. **(D,E)** Transwell assays were used to determine the migration ability of GES-1 cells transfected with lncHEIH or added exosomes to the medium (scale bars = 50 μm). **(F)** The expression levels of EZH2 in GES-1 transfected with lncHEIH or added exosomes to the medium for 48 h. **(G–I)** CCK-8 and Transwell assays were used to determine the proliferation and migration of lncHEIH-overexpressing GES-1 cells transfected with siEZH2-2 (scale bars = 50 μm). *P < 0.05, **P < 0.01, ***P < 0.001.

### The LncHEIH-EZH2 Axis Promotes the Malignant Transformation of Normal Gastric Cells by Stimulating Methylation of the GSDME Promoter

EZH2 has been reported to be an oncogene that generally functions by inhibiting tumor suppressor gene expression (Han Li and Chen, 2015). We analyzed the target genes of EZH2 using Harmonizone website and found 1940 targets from the CHEA Transcription Factor Targets dataset^1^. Then, several well-known tumor suppressor genes related to stem cells in gastric cancer, such as EphB3, E-cadherin, STAT3, P16, PTEN, GSDME, and GSDMB were selected as target genes for the following analysis (Fujii and Ochiai, 2008; Pan et al., 2016; Chen et al., 2017; Gan et al., 2018; Ni et al., 2018; Xu et al., 2018; Li et al., 2020). We determined the expression of these tumor suppressor genes by qRT-PCR when EZH2 was knocked down in lncHEIH-overexpressing cells. The results showed that the transcription levels of PTEN and GSDME were upregulated most significantly (Figure 6A). However, only the expression level of GSDME was affected by lncHEIH, and the inhibition of GSDME expression was reduced after EZH2 interference (Figure 6B). When lncHEIH was overexpressed or exosomes containing lncHEIH were added, downregulated expression of GSDME was observed in normal gastric cells, but no evident change in PTEN was observed (Figure 6C). All of these results suggested that the lncHEIH-EZH2 axis inhibited the expression of GSDME in normal gastric cells. Similarly, we tested whether the downregulation of GSDME participates in the lncHEIH mediated cell malignant transformation. We supplemented lncHEIH-overexpressing GES-1 cells with GSDME, and the abnormalities in cell proliferation and migration were obviously inhibited by GSDME overexpression (Figures 6D–F). These results illustrated that the lncHEIH-EZH2 axis promotes the proliferation and migration of gastric cells by inhibiting GSDME expression.

**FIGURE 6:** The lncHEIH-EZH2 axis promotes malignant transformation of normal gastric cells by stimulating methylation of the GSDME promoter. **(A)** qRT-PCR analysis was used to determine the mRNA levels of EZH2-related tumor suppressor genes when EZH2 was interfered in lncHEIH-overexpressing GES-1 cells. **(B)** Immunoblot analysis of GSDME and PTEN protein levels in lncHEIH-overexpressing cells transfected with siEZH2-2 for 48 h. **(C)** The expression levels of EZH2, GSDME and PTEN in GES-1 transfected with lncHEIH or added exosomes to the medium for 48 h. **(D–F)** CCK-8 and Transwell assays were used to determine the proliferation and migration of lncHEIH-overexpressing GES-1 cells transfected with GSDME (scale bars = 50 μm). **(G)** The promoter deactivation of GSDME caused by EZH2 was reduced when the histone methyltransferase inhibitor GSK126 was added. The results shown are the mean ± SD from three independent experiments. **(H,I)** Methylated bisulfite sequencing PCR analysis. GES-1 cells transfected with EZH2 expression plasmid or empty control plasmid were collected. The methylation level of the GSDME promoter CpG island was detected by bisulfite sequencing PCR. *P < 0.05, **P < 0.01, ***P < 0.001. **(J)** Graphical abstract showing that exosome-delivered lncHEIH promotes gastric cancer progression by upregulating EZH2 and stimulating methylation of the GSDME promoter.

As EZH2 is a methyltransferase, the promoter of GSDME is very sensitive to methylation (Kim et al., 2008; Fujikane et al., 2010). Therefore, we speculated that the downregulation of GSDME might be related to the methylase activity of EZH2. To reveal whether EZH2 acts on the promoter region of GSDME, constructs containing a luciferase reporter and the promoter of GSDME were generated and co-transfected with EZH2 in 293T cells. Reduced luciferase activity was observed when EZH2 was overexpressed (Figure 6G). However, when cells were treated with the histone methyltransferase inhibitor GSK126, the reduced expression of luciferase was rescued (Figure 6G), indicating that EZH2 can act on the promoter region of GSDME. Then, the CpG island of the GSDME promoter was analyzed, and bisulfite sequencing PCR analysis of the GSDME promoter CpG island (chr7:24757597–24757895) was carried out. The results showed that the total methylation level of this CpG island was only 0.6% in the normal gastric cell line GES-1 but increased to 98.1% after overexpression of EZH2 in GES-1 cells (Figures 6H,I). These results suggest that EZH2 could highly methylate the promoter of GSDME, leading to the inhibition of GSDME expression in normal gastric cells.

## Discussion

Over the past decades, the exploration of biomarkers for cancer has been undertaken by multiple researchers (Lee et al., 2019; Lu et al., 2020). Since exosome-delivered lncRNAs can be detected directly from the plasma and sera of patients, they are regarded as potential tumor markers with the advantages of convenient and non-invasive detection. Several lncRNAs have been developed as biomarkers for the detection of cancer at early stages. For example, a high level of lncH19 in serum exosomes was considered to be associated with poor disease prognosis in bladder cancer (Wang et al., 2018). Linc00974, which is involved in the TGF-β-associated pathway, has been identified as a biomarker for HCC diagnosis (Tang et al., 2014). LncRNA 91H and lncCRNDE-h in plasma have been proven as novel biomarkers for the early diagnosis of CRC (Liu et al., 2016; Gao et al., 2018). In addition, lncZFAS1 is also elevated in serum-derived exosomes of gastric cancer (Pan et al., 2017). However, there is no reliable universal tumor marker for gastrointestinal tumors so far.

LncHEIH was first discovered in HCC, in which it was reported to bind EZH2 and regulate the expression of genes promoting tumor progression (Yang et al., 2011). In HCV-related hepatocellular carcinoma, exosome-delivered lncHEIH can enter the bloodstream and be detected in the serum (Zhang et al., 2018). In CRC cells, lncHEIH can promote tumorigenesis by abolishing miRNA-mediated transcriptional repression of Bcl-xL (Cui et al., 2018). In the current study, we found that lncHEIH was increased in gastric cancer. High expression of lncHEIH can affect proliferation and migration *in vitro* and stimulate tumorigenesis of gastric cancer cells and the expansion of gastric CSC in the tumor microenvironment. As a histone lysine *N*-methyltransferase and an oncogenic gene in cancer cells, EZH2 silences many tumor suppressor genes, such as E-cadherin and INK4A/ARF, via canonical H3K27me3 (Hirohito and Hung, 2014; Han Li and Chen, 2015). It also methylates substrates other than H3K27, such as RORα and STAT3 (Lee et al., 2012; Kim et al., 2013). Moreover, upregulated EZH2 plays a crucial role in priming the self-renewal of CSC (Han Li and Chen, 2015). In previous reports, the interaction between lncHEIH and EZH2 has only been found in HCC. Here, we found that lncHEIH can significantly regulate EZH2 expression and promote cancer progression in gastric cancer. Therefore, although the specific regulatory mechanism of lncHEIH and EZH2 still required much more studies, the lncHEIH-EZH2 axis may be a ubiquitous cancer-promoting factor. These results make up for the lack of preceding studies.

Moreover, lncHEIH can be encapsulated by exosomes and then transferred to normal gastric cells. Similarly, lncHEIH entering cells leads to the upregulation of EZH2 in normal gastric cells. At the same time, with the uptake of lncHEIH, the proliferation and migration ability of gastric cells were enhanced. This suggests that exosome-delivered lncHEIH can promote the malignant transformation of normal gastric cells. Moreover, the malignant transformation of cells is closely related to EZH2. As a histone lysine *N*-methyltransferase, EZH2 silences many tumor suppressor genes in cancer cells and promotes the progression of tumor through its methylase activity (Lee et al., 2012; Kim et al., 2013). Here, we further found that the lncHEIH-EZH2 axis promotes the proliferation and migration of gastric cells by inhibiting GSDME expression. The upregulation of EZH2 caused by lncHEIH could substantially increase the methylation level of the GSDME promoter (as illustrated in Figure 6J). GSDME could be specifically cleaved by caspase 3 to generate a gasdermin N-terminal domain which can target the cell membrane, leading to swelling and cell death (Wang et al., 2017). In addition to its roles in necrotic activity, GSDME is a candidate tumor suppressor that is generally downregulated in tumor tissues and cells (Akino et al., 2006). The expression of GSDME suppresses colony formation and cell proliferation in gastric cancer, CRC and melanoma cells (Kim et al., 2008; Rogers et al., 2019). As a previous study reported, the expression of GSDME is downregulated, and such deficiency can be restored when gastric cancer cells are treated with a methyltransferase inhibitor (Akino et al., 2006). Moreover, as a tumor suppressor gene, GSDME has been declared to inhibit tumor progression in breast cancer, gastric cancer and CRC by activating antitumor immunity or inhibiting colony formation and cell proliferation (Zhang et al., 2020). Thus, the increased methylation level of the GSDME promoter regulated by EZH2 may be important for the development of gastric cancer.

Taken together, these observations suggest that lncHEIH is generally upregulated and plays an important role in the development of various gastrointestinal tumors, indicating its potential as a universal biomarker for gastroenteric tumors. Moreover, discovering a suitable EZH2 inhibitor or lncHEIH RNA interfering molecules may provide significant help in the treatment of gastric cancer. Thus, exosome-delivered lncHEIH may be used as a novel target for the treatment of gastric cancer in addition to its diagnostic value.

## Conclusion

This study is the first to report that lncHEIH promotes gastric cancer progression by upregulating the expression of EZH2 and stimulating the methylation of the GSDME promoter. In this process, exosomes successfully transfer the highly expressed oncogene lncHEIH into normal cells to stimulate the expression of EZH2, resulting in high methylation of the GSDME promoter to promote tumorigenesis. This study suggests that lncHEIH is not only a potential universal biomarker for gastroenteric tumors but also a putative target for the treatment of gastric cancer.

## Data Availability Statement

The raw data supporting the conclusions of this article will be made available by the authors, without undue reservation.

## Ethics Statement

The studies involving human participants were reviewed and approved by the Sun Yat-sen University Institutional Animal Care and Use Committee. The patients/participants provided their written informed consent to participate in this study. The animal study was reviewed and approved by the Sun Yat-sen University Institutional Animal Care and Use Committee.

## Author Contributions

YL, KH, SY, and XW performed and analyzed the experiments. XW provided clinical samples. YL, ML, and SY wrote the manuscript. All authors read and approved the manuscript.

## Conflict of Interest

The authors declare that the research was conducted in the absence of any commercial or financial relationships that could be construed as a potential conflict of interest.

## Footnotes

1 http://amp.pharm.mssm.edu/Harmonizome/gene_set/EZH2/CHEA+Transcription+Factor+Targets
